# Efficient Prediction of Missed Clinical Appointment Using Machine Learning

**DOI:** 10.1155/2021/2376391

**Published:** 2021-10-22

**Authors:** Zeeshan Qureshi, Ayesha Maqbool, Alina Mirza, Muhammad Zubair Iqbal, Farkhanda Afzal, Deborah Dormah Kanubala, Tauseef Rana, Mir Yasir Umair, Abdul Wakeel, Said Khalid Shah

**Affiliations:** ^1^CSE, MCS, National University of Sciences and Technology, Islamabad, Pakistan; ^2^DCS, NBC, National University of Sciences and Technology, Islamabad, Pakistan; ^3^DEE, MCS, National University of Sciences and Technology, Islamabad, Pakistan; ^4^ORIC, National University of Modern Languages, Islamabad, Pakistan; ^5^H&BS, MCS, National University of Sciences and Technology, Islamabad, Pakistan; ^6^Academic City University, Accra, Ghana; ^7^CS, University of Science and Technology, Bannu, Pakistan

## Abstract

Public health and its related facilities are crucial for thriving cities and societies. The optimum utilization of health resources saves money and time, but above all, it saves precious lives. It has become even more evident in the present as the pandemic has overstretched the existing medical resources. Specific to patient appointment scheduling, the casual attitude of missing medical appointments (no-show-ups) may cause severe damage to a patient's health. In this paper, with the help of machine learning, we analyze six million plus patient appointment records to predict a patient's behaviors/characteristics by using ten different machine learning algorithms. For this purpose, we first extracted meaningful features from raw data using data cleaning. We applied Synthetic Minority Oversampling Technique (SMOTE), Adaptive Synthetic Sampling Method (Adasyn), and random undersampling (RUS) to balance our data. After balancing, we applied ten different machine learning algorithms, namely, random forest classifier, decision tree, logistic regression, XG Boost, gradient boosting, Adaboost Classifier, Naive Bayes, stochastic gradient descent, multilayer perceptron, and Support Vector Machine. We analyzed these results with the help of six different metrics, i.e., recall, accuracy, precision, F1-score, area under the curve, and mean square error. Our study has achieved 94% recall, 86% accuracy, 83% precision, 87% F1-score, 92% area under the curve, and 0.106 minimum mean square error. Effectiveness of presented data cleaning and feature selection is confirmed by better results in all training algorithms. Notably, recall is greater than 75%, accuracy is greater than 73%, F1-score is more significant than 75%, MSE is lesser than 0.26, and AUC is greater than 74%. The research shows that instead of individual features, combining different features helps make better predictions of a patient's appointment status.

## 1. Introduction

During the COVID-19 pandemic, the world has experienced that the care of critical patients is most strenuous for the health system. Governments have opted for full long-term lockdowns as preventive measures to keep the numbers of urgent care patients low. There are many reasons due to which a patient may reach such a critical state. One of which is not following up with the Primary Care Provider (PCP). The complete treatment of any disease or health issue requires proper treatment and multiple patient visits to PCP. So, PCP needs to plan policies that will provide appropriate alerts/notifications to the patients in a difficult situation and failing to follow up. Mostly, socio and financial challenges lead the patient to miss appointments. Based on the medical specialist review [1], missing appointments cause much more damage than just revenue generation. It affects the care of a patient, patient satisfaction, staff, and overall medical resource utilization. The resource includes valuable time, arrangement of environment for surgery, or any special care suggested to the patient.

Research shows that lowering the rate of missed appointments can improve clinical efficiency and utilization, reduce waste, improve provider satisfaction, and lead to better health outcomes for patients [2]. In this research, we worked on over 6 million records of data. We performed different analyses over it to extract previously unknown and hidden causes and relationships between unique attributes of the patient that lead them not to show up in follow-up appointments. We analyzed unique attributes of patients and applied different algorithms to extract useful features for our analysis. Data we receive at first was not in analyzable form. Using data stored in Electronic Healthcare Record (EHR) systems, we got over six million records that we used in our research to predict which type of patient will miss follow-up appointments (termed as no-show-up appointment in the rest of the article).

Data used for analysis is obtained from thirty-five PCP systems. As per ethics and privacy issues, we have followed guidelines set out under the Health Insurance Portability and Accountability Act (HIPAA), amended by the Health Information Technology for Economic and Clinical Health (HITECH) and Omnibus Final Rule. Therefore, we will only discuss aggregated statistics in the rest of the paper. Protected Health Information (PHI) attributes that create any privacy issue are discarded from feature lists like medical record numbers, patient names, addresses, contact details, and language. The investigated algorithms will take some PHI as inputs to create a useful feature like date of birth to age and then to age range. But outputs and metrics used to optimize and score the algorithms do not use any PHI directly that can cause privacy protection issues.

The motivation of this research is to help healthcare providers make policies so they can find outpatients having a higher risk of chronic disease and having a higher probability of missing their appointments. With the help of this analysis, hospital administration can formulate ways and policies to support the patient in the follow-up of their appointments. Using knowledge of this analysis, the hospital can optimize the utilization of resources, including highly qualified doctors and hospital rooms. Another focus of our research is finding the seasonality/trends of appointments. With the help of this information, hospitals and other healthcare centers can make a necessary plan for seasons having a large number of appointments. Thus, resource utilization can be improved by utilizing our analysis.

In this paper, Section 2 refers to the related work in the field of machine learning, in particular, to no-show-up appointment analysis. In Section 3, we have discussed our technique and process of preparing data for analysis. Then, we discussed methods we applied for predicting missed appointments. In Section 4, we presented the results that we obtain by using the mentioned algorithms.  Section 5 discusses our results by comparing them with existing studies and explaining how our analysis adds value to the field.  Section 6 is the conclusion of our work.

The construction of a good ML model is more of an art than a science. Each model has its features, strengths, and applications. It is essential to distinguish the performance of each model on some standard criteria. In ML, we have four different types of metrics to evaluate the performance of a model: (1) threshold type of discriminator metrics, (2) mean square error (MSE) [3], (3) area under ROC curve (AUC) [4], and (4) hybrid discriminator metric. Davis et al. well drawn detailed comparison of evaluation metrics [5]. It is found that the most commonly used metrics are threshold-type discriminator metrics. Among these, accuracy is considered the most critical measure. But one of the main limitations of accuracy is that it produces less distinctive and less discriminable values [6, 7]. If data classes are imbalanced, an attempt made to analyze data may achieve better accuracy. But that accuracy is not helpful as other metrics like recall, precision, and F1-score values are very low due to poor discrimination of data as mentioned in papers [6, 7]. Therefore, we need the help of different techniques to balance data classes so all metrics give a better result.

Furthermore, it is also powerless in terms of informativeness [8] and less favorable toward minority class instances [8–12]. Informativeness is a characteristic that helps to discriminate how good or bad (informative and noninformative) a solution is. Being less favorable to the minority is a big flaw of accuracy. Solely based on accuracy, one cannot infer that a solution is good or bad. A combination of accuracy with other metrics can give a better understanding of the efficiency of the solution. Other useful features are precision, recall, F1-score, sensitivity (sn), and specificity (sp). While accuracy and recall have a relationship between them [13], by improving one metric, the other is also affected. MSE is used in Supervised Learning Vector Quantization (LVQ) to measure classification performance [14]. AUC is one of the most popular ranking type metrics. The most beneficial characteristic of these metrics is the overall ranking of the performance of the classifier in the multiclass problem [15]. A hybrid discriminator metric is a combination of different threshold type discriminator metrics. Optimized precision [11] and optimized accuracy with recall and precision [16] fall under hybrid metrics. These are evaluation metric criteria based on which solution will be evaluated later in this paper.

While dealing with data, one of the crucial tasks is to deal with imbalance classes of data. Data balancing techniques are used to manipulate data, to have an equal number of records in each class for analysis. For this purpose, the Synthetic Minority Oversampling Technique (SMOTE) algorithm generates excellent results. Using the SMOTE algorithm, the minority class is oversampled by taking each minority class sample and introducing synthetic examples along the line segments joining any/all of the *K*-nearest neighbors [17]. In the case of the imbalance class, improved accuracy can be obtained. But recall and other metrics will show very low values. This indicates poor discrimination in data. The SMOTE algorithm improves results by balancing minority classes. But relying on balanced data using one technique may also lead us toward biased analysis due to the inherent nature of the algorithm. For instance, SMOTE does not handle datasets with all nominal features but handle mixed datasets of continuous and nominal features. [18]. Therefore, its different variations are proposed. To cope up with these issues, we choose two other techniques Adasyn and RUS. So that we can compare differently balanced data rather than relying on a single technique dataset.

## 2. Related Work

At present, there is a scarcity of studies addressing the prediction of no-show-up appointments. Most papers describe the use of one parametric model, for instance, the use of ordinary least square to predict on a given day how many no-show-up appointments will occur. Logistic regression for binary classification is used to predict appointment misses of the patient [19]. Most studies use very few features and apply limited analysis. Few studies developed regression models to predict appointment nonadherence [20, 21]. Some retrospective studies also worked on predicting no-show-up appointments [22]. But that applies to a small dataset of few thousand records.

The most relevant analysis can be seen in the paper of Denney et al. [23]. In this paper, the authors predicted no-show appointments using machine learning algorithms, as the article focused on the effects of missed appointments on revenue, which is a practical application of missed appointment analysis. For this purpose, they focused on the income class category for analysis, which is a significant concern in no-show-up. In this analysis, they used data in millions. They applied analysis of 10 algorithms Adaboost, logistic regression [24], Support Vector Machine (SVM) [25], Naive Bayes [26], stochastic gradient descent [27], extra trees, decision tree, XG Boost, and random forest [28].  Table 1 shows the critical contributions of our work in comparison to other existing studies.

Another paper by AlMuhaideb et al. [29] shows an analysis of no-show appointments through artificial intelligence. In this paper, the authors use a dataset of over a million records. They build predictive models with machine learning algorithm JRip [32] and Hoeffding tree algorithm [33]. In [31], data used is provided by their national health center of authors' country. Five algorithms, random forest, gradient boosting, logistic regression, SVM, and multilayer perceptron, were used [34]. We have adopted the same algorithms as [34]. We further analyzed our results on five different metrics for better evaluation. Mentioned research helps us to identify some of the essential factors to predict the no-show appointments. Mohammadi et al. [30] collected electronic health record (EHR) data and appointment data, including patient, provider, and clinical visit characteristics, over three years. It applied logistic regression, artificial neural network, and Naive Bayes' classifier models to predict missed appointments.

Our work has analyzed similar models with extended five different metrics for better evaluation of the performance model. We have identified important factors to predict the no-show appointments. To get any ML model to work well, good feature selection and better algorithm parameters to create a model are vital tasks. The following are the contributions of our research work:

- Extraction of meaningful attributes based upon entropy and information gain of features
- Analysis and comparison of the performance of three different balancing techniques: SMOTE, Adasyn, and RUS
- Application of ten ML models, namely, random forest classifier, decision tree, logistic regression, XG Boost, gradient boosting, Adaboost Classifier, Naive Bayes, stochastic gradient descent, multilayer perceptron, and Support Vector Machine
- Evaluation of results based on six metrics, i.e., recall, accuracy, precision, F1-score, area under the curve, and minimum mean square error

By considering only recall, the random forest classifier gives us a maximum score. By considering other metrics, the decision tree algorithm gives better results by comparing all balancing techniques.

## 3. Technique and Method Used

In this paper, the data contains about six million records. In raw format, these records are straightforward entries by EHR. From this dataset, features are extracted for analysis using recommended approaches to machine learning. Steps used for analysis are mentioned in the following subsections.

### 3.1. Data Acquisition and Feature Generation

Data obtained for this research is in the transactional form of the SQL Database. Required data is present in different SQL tables. It is separated and dumped into csv file for further analysis. There are two types of appointments that are present in available data. The first one is the closed type, which means the patient appeared in front of PCP and the appointment has been completed by providing any prescription or treatment. The second type is the canceled one, either appointment has been canceled by proper informing to PCPs or it may contain no-show-up data. The difference between canceled and no-show-up is made upon the canceled reason feature. Appointments having a reason for no performance up are considered for our analysis, while the other is kept in the category of show-up even if canceled.

As mentioned earlier, only aggregated PHI data is used for analysis. Initial data is not directly useful for analysis; however, meaningful features are generated from this raw data using feature generations, like the feature of age range which is created with the help of date of birth. Similarly, the appointment season feature is obtained with the help of the appointment date characteristic. Individual features like appointment creation date are relevant for analysis. But by combining these, a better feature is obtained like the difference between the date of appointment and creation date giving us an appointment to create the difference. This information helps us to predict that if a difference of appointment is that more than 2 months, the patient is less likely to show up for an appointment. These are just examples; numerous features can be generated using the synthetic generation of features [35]. In Table 2, we provided a list of all useful features that are either individual or formed by a combination of attributes.

By generating many features, there is a need to select the most relevant features useful for predicting no-show-up predictions. For this purpose, we used information gain [36]. It is a useful technique to predict the relevancy of data as it is adopted by many researchers [37–39]. Based upon the information, the characteristic sequence of relevant features is given in Table 3. Table 3 depicts the procedure type feature, which tells us the type of procedure, e.g., angiogram fistula and clinic office visit. There are about 30 plus different types of races available in our data, which contribute better to analysis. Civil status tells about the marital status of the patient. Attribute appointment creating a difference (number of days between the creation of appointment and the actual date of appointment) has a significant influence on predictions. But that attribute was given in the number of days which our models do not readily support. We divided description categories: 1 week, 2 weeks, 3 weeks, 1 month, 2 months, 3 months, 4 months, 5 months, 6 months, 7 months, 8 months, 9 months, 10 months, 11 months, 1 year, 2 years, 3 years, 4 years, and 5 years. The age range feature is also formed by seven categories of patients, which are below 17, 18 to 29, 30 to 39, 40 to 49, 50 to 59, 60 to 69, and 70 onward. The feature appointment season is created by finding months in which appointment has been made. In the current scenario, it is kept from January to December. Sex attribute tells whether the patient is male, female, or unknown. But by checking information gain, it is observed that this feature contributes to prediction at a very low level. In the dataset, the oldest appointment date is 10/10/2007, and the latest appointment is of date 02/28/2022. Future appointments are also present in the system whose appointment status is pending. For the current analysis, pending status appointments are ignored.

### 3.2. Data Cleaning

The original data had many empty values and required filtering. Empty values in each feature are analyzed carefully. Available data have some empty values in canceled appointments. But data had an additional modified date feature. The modified date is change in appointment date, which also indicates no-show-up. Once an appointment has been canceled, no further changes can be made to that appointment. So, those empty values are filled with the modified date.

Data used for analysis is obtained by a different source of software. Some of them explicitly store cancel date along with the reason. Some of them just store cancel reason. For the second case, the last modified date is the one for which the modified date is considered a canceled date, because once an appointment is canceled, no further action is performed on that one. So in these cases, the cancel date was extracted from reason and modified date. Some features have no entries and lack reference to any other attribute. Therefore, these entries were discarded. The civil status attribute also has almost five to six different types of values which are not on large counts. These are converted into three different kinds of categories alone, couple, and unknown. In the alone category, single people, divorced, or widowed are kept. While in the couple category, married people are held for analysis. The third category is maintained for those whose civil status is unknown or not mentioned in the record. Table 3 depicts the useful features acquired after proper cleaning. These features helped us to predict better results for the no-show-up final result.

### 3.3. Data Exploration

Before applying models to data for analysis, it is required to explore data in detail to evaluate better results obtained by analysis. Data exploration's first task is to determine how many records we have for show or no-show-up appointments from our data. A clear comparison of the show and no-show-up data can be observed in Figure 1, which shows show and no-show appointments on the *x*-axis and appointment count on the *y*-axis.

Figure 2 illustrates the comparison of patients' appointments with respect to age. Similarly, Figure 3 shows the gender-wise distribution of show and no-show-up appointments. Table 2 depicts the most relevant feature, procedure type, other than age and gender. The pie chart in Figure 4 reveals the different types of procedures in terms of percentage. In this figure, procedure type 0 shows records having an unknown value. But as mentioned in Section 3.2, values that lack valuable reference are ignored for analysis. So, procedure type 0 is discarded for further analysis in this paper.

### 3.4. Balancing Data

Data was cleaned and prepared for use in the analysis. Figures 1–3 depict that data have an imbalance class in nature. In such case, algorithms will tend to predict show-up appointments with greater accuracy. But this prediction is not very good as other metric scores less with such data. To address imbalance data, various techniques were used in literature [23, 40, 41]. In our work, we have adopted the following three techniques to balance classes.

#### 3.4.1. Synthetic Minority Oversampling Technique (SMOTE)

Introduced by Chawla et al. [17] and used by Denney et al. [23] for balancing medical data, SMOTE is proved to be a good approach to balance the classes. The core idea of this technique is to use the undersample of the majority class and the oversample of the minority class. Oversampling is done by introducing synthetic examples along the segment joining any/all of *k* minority class nearest neighbors. These new features are added in feature space, which is then considered again in the next iterations. This process keeps on repeating until a balanced dataset having equal distributed samples is formed.

#### 3.4.2. Adaptive Synthetic Sampling Method (Adasyn)

The core of this technique is similar to SMOTE for the generation of minority class elements. But here, density distribution is considered for synthetic samples, while in SMOTE, uniform weight for minority points is used. Haibo et al. [40] suggest two benefits of using Adasyn:

1. It reduces bias introduced by the class imbalance
2. It adaptively shifts the classification decision boundary toward the complex examples

#### 3.4.3. Random Undersampling (RUS)

We have two approaches to address oversampling of the majority class and the undersampling of the minority class. Drummond et al. [41] analyzed the benefits of random undersampling in different scenarios. Random undersampling is a simple technique that has proven beneficial in balancing data [42]. Samples of majority classes are reduced to equate minority class samples. In this way, equal samples are considered for analysis. Keeping in view the advantages of its simplicity, for analyzing our data, we considered the random undersampling technique.

Figure 5 shows the actual distribution of data, whereas Figure 6 illustrates the distribution after applying these techniques.

### 3.5. Methods Used

In this paper, ten different algorithms are used to no-show.

1. Decision tree
2. Logistic regression
3. Naive Bayes
4. Random forest classifier
5. Adaboost Classifier
6. Support Vector Machine (SVM)
7. XG Boost
8. Gradient boosting
9. Stochastic gradient descent (SGD)
10. Multilayer perceptron

Different parameters are required to be prearranged for these algorithms to perform better. In our study, we ran a different variation and combination of parameters to achieve improved results. We established that not all parameters work best even after cleaning data. It is well known that the appropriate selection of parameters and input data plays an essential role in improved results [43, 44]. In random forest classifier and stochastic gradient descent (which gives results in continuous form), results obtained are in decimal based on their probability to be a show or no-show-up. A threshold is set to be 0.6. The values greater than 0.6 were considered 1, and below 0.6 were referred to as 0.

## 4. Evaluation of Results

Algorithms mentioned in Section 3.5 are applied to the dataset, and models are generated using the holdout technique [45]. Holdout is a useful machine learning technique used to analyze a large dataset. Using this technique, a small chunk of data with random record selection is considered in measuring efficiency of the algorithm while remaining data is used to train the algorithm.

In our case, the data has over 6 million entries. Thus, holdout is used to evaluate models generated using selected algorithms. The best practice of 70-30 is utilized for generating a model where 70% data is preserved for training on which model is developed, and 30% data is kept for testing performance of the algorithm. There are different types of techniques that can be applied to distribute data in training and testing parts like cross-validation and 10-fold cross-validation technique. But the holdout technique is the simplest and most useful.

Data analyzed in Table 4 is based on SMOTE. Threshold type discriminator metrics and evaluation of algorithm analysis data are presented in Figure 3. On threshold type discriminator evaluation, the best results in terms of accuracy alone are obtained by the logistic regression. But by keeping in view other attributes, improved results are obtained, i.e., accuracy, 74% precision, 82.26% F1-score, and best of all recall 91%. Recall is considered the best criteria to evaluate the performance of any algorithm. The random forest classifier gives the best recall of no-show predictions. The evaluation of proposed models based on mean square errors and the area under the curve is shown in Table 5. It can be seen that minimum mean square error, i.e., 0.1069, and better area under the curve, i.e., 92.09%, are obtained by the random forest classifier. So based on statistics, we can conclude that random forest performed better on data balanced by SMOTE. Hybrid discriminator metric values are dependent on a combination of threshold discriminator values. The good discriminator values give better metrics of hybrid discriminators [5].

Evaluations shown in Table 6 are based on data balanced by Adasyn. Threshold type discriminator metric results are presented in Table 6. Based on these values, the best result bases upon recall alone is obtained by random forest. But keeping in view other attributes, the decision tree shows better results having 85.03% accuracy, 81% precision, 86% F1-score, and 90% recall. Considering only recall, the random forest gives better results while the decision tree outperforms in other metrics. The evaluation analysis of proposed models based on mean square errors and area under the curve is shown in Table 7. According to that, the decision tree algorithm obtains minimum mean square error, i.e., 0.15, and better area under the curve, i.e., 85.03%. Moreover, in Table 6 and the show-no-show Adasyn appointment prediction evaluation by MSE and AUC statistics, it can be concluded that the decision tree classifier performed better on data balanced by the Adasyn technique.

Data analyzed in Table 8 is based on data balanced by technique RUS. Based on threshold type discriminator metrics, the best results in terms of recall are obtained by random forest, i.e., 94%. But keeping in view other attributes, better results are obtained by the decision tree having 86.5% accuracy, 83% precision, 87% F1-score, and 92% recall. Considering only the recall attribute, the random forest outperforms, while the decision tree performs in other metrics. The evaluation results of proposed models based on mean square errors and the area under the curve are shown in Table 9. According to that, minimum mean square error, i.e., 0.135, and better area under the curve, i.e., 86.5%, are obtained by the decision tree. It can conclude by considering statistics that the decision tree classifier performed better on data balanced by RUS technique.

## 5. Discussion

Based on the result mentioned in Section 3, the following key findings are presented. By referring to research [3, 46], it can be observed that the smaller mean square error (MSE) gives a better prediction. Similarly, study [4] says that the more the value of AUC, the more improved the result. Keeping in view the results given in Table 5, it is concluded that the random forest classifier performs better on the given dataset with the lowest MSE value of 0.1069 and 92.09% AUC value. Show-no-show RUS appointment prediction results evaluated by MSE and AUC are often used to measure the performance of models. Random forest and decision tree performed better in all metrics. From the summarized results of Table 10, 85.26% accuracy from the random forest using SMOTE, Adasyn, and RUS is achieved. The recall is 94% provided by RUS in random forests. F1-score is 86.25% provided by SMOTE under random forest. Mean square error is minimum in SMOTE, i.e., 0.1069 under random forest, while the area under the curve is maximum given by SMOTE 92.09% under random forest. So, out of six metrics, three indicate that RUS balancing technique gives better results, while four indicate that SMOTE is better for the random forest. Similarly, the decision tree's statistics against SMOTE, Adasyn, and RUS are also analyzed. We attained the best accuracy under RUS, i.e., 85.5%; best precision under RUS, i.e., 83%; best recall 92% under RUS; best F1-score 87% under RUS; minimum MSE 0.1285 under SMOTE; and best AUC 87.13% under SMOTE. So, based on that, four out of six metrics indicate that the RUS technique is better, while two out of six metrics favor SMOTE balancing technique. Based on these discussions, we can say that RUS technique for balancing data performs better.

By considering only recall, the random forest classifier gives us a maximum score of 94% with RUS balancing technique. By considering other metrics, the decision tree algorithm gives better results by comparing all balancing techniques. Furthermore, different models also performed well on the given data as their value also improved to more than 55% under all balancing techniques. While referring to these results with other research [23, 29, 31], it can be observed that a better available dataset, better cleaning of data, and good feature selection improve the prediction result of no-show. Another critical factor is that only one metric cannot help categorize the model as good or bad. All values of metrics confirm this argument, that this work adds value to research.

## 6. Conclusion

This study has used 3 different balancing techniques to balance the dataset. The paper presents in detail an explanation of data along with an analysis of useful features for analysis. We have analyzed ten different algorithms with the help of six different types of metrics. Furthermore, we achieve better metric values with our data balancing and feature inclusion technique. Based on the results of this paper, it is validated that only one metric is not enough to tell about model performance. There is a need to evaluate models' performance from multiple metrics. Moreover, balancing techniques can also make a difference in results. The RUS balancing technique and decision tree algorithm are the best options for analyzing whether a patient will show or miss an appointment. Feature selection is a key to get better results like information gain. We have found that features, title, procedure type, races, civil status, create difference, and age range are more effective in getting better predictions. Six different types of metrics achieve improved results than mentioned in the literature. Furthermore, it is verified that the random forest classifier, decision tree, logistic regression, XG Boost, and gradient boosting performed very well, having recall greater than 75%, an accuracy greater than 73%, and F1-score greater than 75%.

## Figures and Tables

**Figure 1:** Comparison of show and no-show appointments.

**Figure 2:** Age-wise comparison of show and no-show appointments.

**Figure 3:** Gender-wise comparison of show and no-show appointments.

**Figure 4:** Procedure-wise distribution of data.

**Figure 5:** Percentage-wise show and no-show distribution of data.

**Figure 6:** Percentage-wise show and no-show distribution after applying SMOTE.

**Table 1:** Comparison to existing research.

Studies	Data	Algorithm	Evaluation method	Performance	
Denney et al. [23]	7 million	Ada, LR, SVM, NB, SGD, ET, DT, XG, RF	Average recall	68% recall	Existing model with results
AlMuhaideb et al. [29]	1.1 million	JRip, Hoeffding trees, LR, MP, NB	Accuracy, AUC	77.13% accuracy, 0.86 AUC	
Mohammadi et al. [30]	74 thousand	LR, MP, NB	Accuracy, AUC	82% accuracy, 0.86 AUC	
Daghistani et al. [31]	201 million	RF, GB, LR, SVM, MP	Accuracy, precision, recall, F1 measure, AUC	79% accuracy, 77% precision, 79% recall, 76% *F* score, 0.81 AUC	
Our model	6 million	Ada, LR, SVM, NB, SGD, XG, DT, GB, RF, MP	Accuracy, precision, recall, F1 measure, AUC, MSE	86.5% accuracy, 83% precision, 94% recall, 87% *F* score, 0.92 AUC, 0.1069 MSE	Proposed model with result

**Table 2:** Useful features.

Name	Type	Range	Description
Date of birth	Input	mm/dd/yyyy	Date of birth of patient
Race	Input	Like Asian, African, white	Race of patient
Sex	Input	Male/female/other	Sex of patient
Civil status	Input	Single, married, divorced, separated, widowed	Civil status
Admit	Input	Textual format	Reason of admission
Date of appointment	Input	mm/dd/yyyy date	Date of appointment
Status of appointment	Input	Pending, closed, canceled	Status of appointment
Cancel date	Input	mm/dd/yyyy date	Canceling appointment date
Cancel reason	Input	No-show-up, death, rescheduled, out of city	Canceling appointment reason
Create time	Input	Time stamp format	Time at which database entry record was inserted
Modified time	Input	Time stamp format	Time at which database entry record was modified
Procedure type	Input	Like ultrasound, office visit see table	In which procedure patient booked appointment
Patient age	Generated	Numeric	Created by date of birth
Age range	Generated	From age category	Created by patient age feature
Create Appt difference	Generated	No of days	Created by taking difference of appointment date and create time
Appointment season	Generated	Month of year	Created with the help of appointment date
Cancel difference	Generated	No. of days	Created by taking difference of cancel date and appointment date

**Table 3:** List of relevant features to predict appointment status.

Relevance	Feature name	Information gain values
1	Procedure type	0.0736
2	Race category	0.04305
3	Civil status	0.019836
4	Create difference category	0.019534
5	Age range	0.000890
6	Appointment season	0.000375
7	Sex	0.0001323

**Table 4:** Threshold discriminative metric evaluation for show and no-show appointment prediction.

Algorithm	Accuracy	Precision	Recall	F1-score
Random forest	84.96%	80%	93%	86.25%
Decision tree	85.18%	82%	90%	86.42%
Logistic regression	85.35%	83%	89%	86.18%
XG Boost	76.69%	80%	83%	81.44%
Gradient boosting	73.53%	76%	77%	77.32%
Adaboost	70.46%	74%	72%	73.17%
SVM	67.09%	69%	74%	72.15%
Naive Bayes	63.98%	66%	70%	68.44%
SGD	67.14%	60%	84%	70.18%
Multilayer perceptron	80.93%	64%	77%	70.52%

**Table 5:** Show and no-show appointment prediction result by mean square error and AUC.

Algorithm	MSE	AUC
Random forest	0.1069	92.09%
Decision tree	0.1285	87.13%
Logistic regression	0.1273	87.25%
XG Boost	0.1906	80.92%
Gradient boosting	0.2330	76.69%
Adaboost	0.2646	73.53%
SVM	0.2953	70.45%
Naive Bayes	0.3277	67.21%
SGD	17.71	55.47%
Multilayer perceptron	0.3282	67.14%

**Table 6:** Show and no-show Adasyn appointment prediction result evaluation by threshold discriminative metrics.

Algorithm	Accuracy	Precision	Recall	F1-score
Random forest	85.26%	78%	93%	85%
Decision tree	86.50%	81%	90%	86%
Logistic regression	64.77%	66%	66%	66%
XG Boost	79.12%	77%	81%	79%
Gradient boosting	75.69%	74%	75%	75%
Adaboost	71.90%	72%	70%	71%
Naive Bayes	65.37%	65%	68%	67%
SGD	60.96%	59%	83%	69%
Multilayer perceptron	63.61%	65%	69%	67%
SVM	68.58%	67%	72%	70%

**Table 7:** Show and no-show Adasyn appointment prediction result by mean square error and AUC.

Algorithm	MSE	AUC
Random forest	0.16	83.26%
Decision tree	0.15	85.03%
Logistic regression	0.334	66.51%
XG Boost	0.21	78.43%
Gradient boosting	0.255	74.46%
Adaboost	0.279	71.98%
Naive Bayes	0.338	66.20%
SGD	0.339	63.49%
Multilayer perceptron	0.3408	65.94%
SVM	0.28	68.90%

**Table 8:** Show-no-show RUS appointment prediction result evaluation by threshold discriminative metrics.

Algorithm	Accuracy	Precision	Recall	F1-score
Random forest	85.26%	80%	94%	86%
Decision tree	86.50%	83%	92%	87%
Logistic regression	64.77%	65%	65%	65%
XG Boost	79.12%	78%	81%	79%
Gradient boosting	75.69%	76%	76%	76%
Adaboost	71.90%	74%	67%	70%
Naive Bayes	65.37%	65%	68%	66%
SGD	60.96%	58%	83%	68.18%
Multilayer perceptron	63.61%	59%	88%	71%
SVM	68.58%	68%	71%	69%

**Table 9:** Show-no-show RUS appointment prediction result evaluation by mean square error and AUC.

Algorithm	MSE	AUC
Random forest	0.1473	85.26%
Decision tree	0.135	86.50%
Logistic regression	0.352	64.77%
XG Boost	0.208	79.12%
Gradient boosting	0.243	75.68%
Adaboost	0.281	71.9%
Naive Bayes	0.346.	65.37%
SGD	0.3546	60.96%
Multilayer perceptron	0.3648	63.62%
SVM	0.26.	68.58%

**Table 10:** Comparison of all balanced analyzed data against random forest and decision tree.

Measures	Algorithms	Random forest (%)	Decision tree
Accuracy (%)	SM-AD-RUS	84.96-83.17-85.26	85.18-85.03-86.50
Precision (%)	SM-AD-RUS	80-78-80	82-81-83
Recall (%)	SM-AD-RUS	93-93-94	90-90-92
F1-score (%)	SM-AD-RUS	86.25-85-86	86.42-86-87
MSE	SM-AD-RUS	0.1069-0.16-0.1473	0.1285-0.15-0.135
AUC (%)	SM-AD-RUS	92.09-83.26-85.26	87.13-85.03-86.50

## Data Availability

There is no data available to support the study.

## References

[1] Marbouh D., Khaleel I., al Shanqiti K. (2020). Evaluating the impact of patient no-shows on service quality. *Risk Management and Healthcare Policy*.

[2] Molfenter T. (2013). Reducing appointment no-shows: going from theory to practice. *Substance Use & Misuse*.

[3] Allen D. M. (1971). Mean square error of prediction as a criterion for selecting variables. *Techno Metrics*.

[4] Myerson J., Green L., Warusawitharana M. (2001). Area under the curve as a measure of discounting. *Journal of the Experimental Analysis of Behavior*.

[5] Davis J. V., Kulis B., Jain P., Sra S., Dhillon I. S. Information-theoretic metric learning.

[6] Huang J., Ling C. X. (2007). *Constructing New and Better Evaluation Measures for Machine Learning*.

[7] Rakotomamonjy A. (2004). *Optimizing Area under Roc Curve with SVMs*.

[8] Mac Kay D. J., Mac Kay D. J. (2003). *Information Theory, Inference and Learning Algorithms*.

[9] García S., Herrera F. Evolutionary training set selection to optimize c4. 5 in imbalanced problems.

[10] Hossin M., Sulaiman M., Mustapha A., Mustapha N., Rahmat R. A hybrid evaluation metric for optimizing classifier.

[11] Ranawana R., Palade V. Optimized precision-a new measure for classifier performance evaluation.

[12] Wilson S. W. (2000). Mining oblique data with XCS. *International Workshop on Learning Classifier Systems*.

[13] Buckland M., Gey F. (1994). The relationship between recall and precision. *Journal of the American Society for Information Science*.

[14] Kohonen T. (2012). *Self-Organizing Maps, vol. 30*.

[15] Hand D. J., Till R. J. (2001). A simple generalisation of the area under the ROC curve for multiple class classification problems. *Machine Learning*.

[16] Hossin M., Sulaiman M. N. (2015). A review on evaluation metrics for data classification evaluations. *International Journal of Data Mining & Knowledge Management Process*.

[17] Chawla N. V., Bowyer K. W., Hall L. O., Kegelmeyer W. P. (2002). SMOTE: synthetic minority over-sampling technique. *Journal of Artificial Intelligence Research*.

[18] Ganganwar V. (2012). An overview of classification algorithms for imbalanced datasets. *International Journal of Emerging Technology and Advanced Engineering*.

[19] Ding X., Gellad Z. F., Mather C. (2018). Designing risk prediction models for ambulatory no-shows across different specialties and clinics. *Journal of the American Medical Informatics Association*.

[20] Huang Y., Hanauer D. A. (2014). Patient no-show predictive model development using multiple data sources for an effective overbooking approach. *Applied Clinical Informatics*.

[21] Huang Y., Zuniga P. (2014). Effective cancellation policy to reduce the negative impact of patient no-show. *Journal of the Operational Research Society*.

[22] Kaplan-Lewis E., Percac-Lima S. (2013). No-show to primary care appointments. *Journal of Primary Care & Community Health*.

[23] Denney J., Coyne S., Rafiqi S. (2019). Machine learning predictions of no-show appointments in a primary care setting. *SMU Data Science Review*.

[24] Cramer J. S. (2002). *The Origins of Logistic Regression*.

[25] Dinov I. D. (2016). Methodological challenges and analytic opportunities for modeling and interpreting big healthcare data. *Gigascience*.

[26] Rish I. An empirical study of the naive Bayes classifier.

[27] Friedman J. H. (2002). Stochastic gradient boosting. *Computational Statistics & Data Analysis*.

[28] Rodriguez-Galiano V. F., Ghimire B., Rogan J., Chica-Olmo M., Rigol-Sanchez J. P. (2012). An assessment of the effectiveness of a random forest classifier for land- cover classification. *ISPRS Journal of Photogrammetry and Remote Sensing*.

[29] AlMuhaideb S., Alswailem O., Alsubaie N., Ferwana I., Alnajem A. (2019). Prediction of hospital no-show appointments through artificial intelligence algorithms. *Annals of Saudi Medicine*.

[30] Mohammadi I., Wu H., Turkcan A., Toscos T., Doebbeling B. N. (2018). Data analytics and modeling for appointment no-show in community health centers. *Journal of Primary Care & Community Health*.

[31] Daghistani T., AlGhamdi H., Alshammari R., AlHazme R. H. (2020). Predictors of outpatients’ no-show: big data analytics using Apache Spark. *Journal of Big Data*.

[32] Cohen W. W. Fast effective rule induction.

[33] Hulten G., Spencer L., Domingos P. Mining time-changing data streams.

[34] Baitharu T. R., Pani S. K. (2016). Analysis of data mining techniques for healthcare decision support system using liver disorder dataset. *Procedia Computer Science*.

[35] Zięba M., Tomczak S. K., Tomczak J. M. (2016). Ensemble boosted trees with synthetic features generation in application to bankruptcy prediction. *Expert Systems with Applications*.

[36] Azhagusundari B., Thanamani A. S. (2013). Feature selection based on information gain. *International Journal of Innovative Technology and Exploring Engineering*.

[37] Uguz H. (2011). A two-stage feature selection method for text categorization by using information gain, principal component analysis and genetic algorithm. *Knowledge-Based Systems*.

[38] Stachniss C., Grisetti G., Burgard W. (2005). Information gain-based exploration using rao-blackwellized particle filters. *Robotics: Science and Systems*.

[39] Nelson J. D. (2005). Finding useful questions: on Bayesian diagnosticity, probability, impact, and information gain. *Psychological Review*.

[40] He H., Yang B., Garcia E. A., Li S. ADASYN: adaptive synthetic sampling approach for imbalanced learning.

[41] Drummond C., Holte R. C. C4. 5, class imbalance, and cost sensitivity: why under-sampling beats over-sampling.

[42] Seiffert C., Khoshgoftaar T. M., Van Hulse J., Folleco A. (2014). An empirical study of the classification performance of learners on imbalanced and noisy software quality data. *Information Sciences*.

[43] Gardner M. W., Dorling S. (1998). Artificial neural networks (the multilayer perceptron)--a review of applications in the atmospheric sciences. *Atmospheric Environment*.

[44] Biau G., Scornet E. (2016). A random forest guided tour. *Test*.

[45] Scruggs P. W., Beveridge S. K., Eisenman P. A., Watson D. L., Shultz B. B., Ransdell L. B. (2003). Quantifying physical activity via pedometry in elementary physical education. *Medicine and Science in Sports and Exercise*.

[46] Willmott C. J., Matsuura K. (2005). Advantages of the mean absolute error (MAE) over the root mean square error (RMSE) in assessing average model performance. *Climate Research*.

